The article "Identification of Oxidative Stress-Associated Molecular Subtypes and Signature for Predicting Survival Outcome of Cervical Squamous Cell Carcinoma" was retracted in 2023. Reasons: suspected computer-generated content; unreliable results or conclusions; concerns about the data; concerns about the results or conclusions.

# Identification of Oxidative Stress-Associated Molecular Subtypes and Signature for Predicting Survival Outcome of Cervical Squamous Cell Carcinoma

**DOI:** 10.1155/2022/1056825

**Published:** 2022-10-03

**Authors:** Lei Wang, Hui Qu, Xiaolin Ma, Xiaomei Liu

**Affiliations:** Department of Obstetrics and Gynecology, Shengjing Hospital of China Medical University, Shenyang City, China 110004

## Abstract

**Background:**

Cervical squamous cell carcinoma (CESC) is the gynecologic malignancy with high incidence rate and high mortality rate. Oxidative stress participates in gene regulation and malignant tumor progression, including CESC.

**Methods:**

RNA-seq, clinical information, and genomic mutation were from The Cancer Genome Atlas- (TCGA-) CESC and GSE44001 datasets. Oxidative stress-related genes were obtained from the gene set enrichment analysis (GSEA) website. ConsensusClusterPlus was used for clustering, which was assessed by the Kaplan-Meier (KM) survival curve analysis, mutation analysis, immunocharacteristic analysis, and therapy. Prognostic signatures were built by combining weighted correlation network analysis (WGCNA), least absolute shrinkage and selection operator (LASSO) algorithm, and stepAIC. The prognostic power of this model was evaluated using the KM survival curve analysis, receiver operating characteristic (ROC) curve analysis, nomogram, and decision curve analysis (DCA).

**Results:**

218 of the 291 CESC cases (74.91%) presented oxidative stress-related gene mutation, especially FBXW7. Three clusters were determined based on oxidative stress-related genes, among which cluster 3 (C3) presented low-frequency mutation and hyperimmune state and was sensitive to immunotherapy. This research developed a 5-gene oxidative stress-related prognostic signature and a RiskScore model. As shown by ROC analysis, in the TCGA and GSE44001 datasets, the RiskScore model showed a high prediction accuracy for 1-, 3-, and 5-year CESC overall survival. High RiskScore was associated with enhanced immune status. The nomogram model was greatly predictive of the overall survival of CESC patients.

**Conclusion:**

Our prognostic model was based on oxidative stress-related genes in CESC, potentially aids in CESC prognosis, and provides potential targets against CESC.

## 1. Introduction

Cervical cancer is one of the most common cancers in women and, unlike in developed countries, has a high death rate in developing countries [1–4]. Cervical cancer cases include cervical adenosquamous cell carcinoma, cervical adenocarcinoma, and cervical squamous cell carcinoma (CESC). CESC is the most common type that accounts for more than 80% of all cervical cancer cases [5]. HPV infection is a pathogenic factor of cervical cancer and other cancers, but its mechanism is still unclear [6]. At the same time, some studies have shown that not all HPV infections lead to cervical cancer, which suggested that in addition to HPV infection, cervical cancer also involves other factors such as genetics and environment [7, 8]. In the 30 years since the cervical cancer screening programme was introduced, both cervical cancer incidence and death rates have fallen by more than 50% [9, 10]. The 5-year survival rate of patients with early CESC is 91.5%, while the 5-year survival rate of patients with recurrent and metastatic cervical squamous cell carcinoma is only 16.5%, and about 13% of patients with cervical squamous cell carcinoma are initially diagnosed as advanced [11]. Lymph node metastasis is a poor prognostic factor [12]. Metastatic or recurrent, node-positive cervical squamous cell carcinoma still has a poor prognosis [11]. Therefore, it is of great theoretical significance and clinical application value to study the pathogenesis of CESC from the molecular level and find specific molecular targets related to cervical squamous cell carcinoma.

A common feature of various complex pathophysiological mechanisms of cancer is the increased utilization of reactive oxygen species (ROS), also known as oxidative stress. Low levels of ROS can be used as second messengers and are involved in various cellular physiological activities, such as signal transduction, apoptosis, senescence, cell proliferation, and migration. Instead, high levels of ROS are thought to be contributing factors to many diseases, including cancer, aging, neurodegenerative diseases, diabetes, cardiovascular disease, stroke, and asthma [13, 14]. However, sustained high levels can cause oxidative damage to cells [15]. The imbalance between ROS and endogenous antioxidant species leads to oxidative stress [16]. Oxidative stress can cause cell death, including apoptosis, depending on its intensity [17].

In this study, transcriptome and clinicopathological and overall survival information for CESC were collected from The Cancer Genome Atlas (TCGA) database. We also collected genes associated with oxidative stress from GSEA. ConsensusClusterPlus method was used to identify molecular subtypes associated with oxidative stress. Then, a prognostic evaluation model for CESC was established based on oxidative stress-related genes. The area under receiver operating characteristic (ROC) curve (AUC), KM survival curve, nomogram, and decision curve analysis (DCA) were used to verify the clinical application potential of the model.

## 2. Material and Methods

### 2.1. Raw Data

RNA-seq data, clinical information, and single-nucleotide variant (SNV) were acquired from TCGA-CESC dataset and GSE44001 dataset. Samples with clinical information, survival time, and status were retained. Waterfall plot was generated to explore the detailed SNV characteristics between molecular subtypes via “mutect 2” function in R software. The clinical information of TCGA-CESC and GSE44001 datasets was listed in Table 1.

OXIDATIVE_STRESS pathways and corresponding oxidative stress genes were obtained from the GSEA website (http://www.gsea-msigdb.org/gsea/index.jsp).

### 2.2. Cluster Analysis

As per the standards of *P* < 0.05, oxidative stress-related genes with prognosis of CESC were determined via univariate Cox survival analysis using coxph function of R package. Then, molecular subtypes were performed separately for TCGA-CESC dataset samples via the ConsensusClusterPlus 1.52.0 [18]. Pam arithmetic and “pearson” distance were utilized to complete 500 bootstraps with every bootstrap having specimens (≥80%) of TCGA-CESC dataset. Cluster number *k* was between 2 and 10, and the optimum *k* was identified as per cumulative distribution function (CDF) and AUC. Survival curves (KM curves) between molecular subtypes were then analyzed for difference. In addition, differences in the distribution of clinical characteristics between molecular subtypes were compared, and a chi-square test was completed, and *P* < 0.05 had significance on statistics.

### 2.3. Gene Set Enrichment Analysis

GSEA (http://software.broadinstitute.org/gsea/index.jsp) was performed to identify hallmarks of the samples of oxidative stress-related gene mutations compared with the nonmutated samples.

### 2.4. Microenvironment Cell Population-Counter (MCP-Counter)

The abundance of immune-infiltrating cells, eight immune populations (cytotoxic lymphocytes, CD8+ T cells, neutrophils, monocytic lineage, T cells, B lineages, natural killer cells, and myeloid dendritic cells), and two stromal populations (fibroblasts and endothelial cells) from the samples were assessed using MCP-counter.

### 2.5. Single-Sample GSEA

The ssGSEA was used to evaluate the infiltration level of the 28 immune cells [19] using GSVA of R package. ssGSEA score was transformed into uniform distribution (between 0 and 1).

### 2.6. Estimate

R software ESTIMATE arithmetic [20] was utilized to compute overall stroma level (StromalScore), the immunocyte infiltration (ImmuneScore), and the combination (ESTIMATEScore) of sufferers in the TCGA-CESC cohort using Wilcox.test analysis to determine difference.

### 2.7. Immunotherapy

The expression levels of the 21 immune checkpoint genes, which from HigsAtlas [21], were determined. Tumor immune dysfunction and exclusion (TIDE) [22, 23] (http://tide.dfci.harvard.edu/) is a calculation framework designed to assess the potential of cancer immunoescape from the genetic expression profiles of tumor specimens. TIDE was used to predict sample responses in the TCGA-CESC datasets and to compare the proportion of treatment responses in different subtypes, as well as TIDE scores. pRRophetic [24] was used to predict the sensitivity of cisplatin, erlotinib, sunitinib, paclitaxel, sorafenib, and crizotinib to IC_50_.

### 2.8. Weighted Correlation Network Analysis (WGCNA)

The TCGA-CESC dataset was applied to separate molecular subtype-related gene modules in the R software package WGCNA [25]. Specifically, the samples were firstly clustered, and the coexpression modules were screened. When log(*k*) of the node showing connection degree of *K* showed a negative correlation with log(*P*(*k*)) of its occurrence probability and the correlation coefficient was greater than 0.85, this indicated that the coexpression network complied with the scale-free network. Further, the gene expression similarity matrix was converted into an adjacency matrix. *β* is a soft-thresholding parameter and represents Pearson's correlation coefficient for each pair of genes [26]. With topological overlap measure (TOM), average linkage level clustering method was employed to cluster genes. In each gene network, the minimum number of genes module was 150. After using dynamic clipping method to determine gene modules, the eigengenes of each module were calculated in turn, followed by conducting cluster analysis on these modules. Using height = 0.25, deepSplit =2, and minModuleSize = 150, close modules were integrated into new modules. Grey module was a set of genes that cannot be combined into the rest of other modules.

The correlation analysis of molecular subtypes and modules, as well as enrichment analysis of molecular subtypes, was analyzed to identify hub module.

### 2.9. Construction of a Prognostic Model for CESC

TCGA-CESC dataset samples were divided into training dataset and test dataset as 1 : 1. In TCGA training dataset, as per the standards of *P* < 0.01, genes, which from above screened hub module, with prognosis of CESC were determined via univariate Cox survival analysis using coxph function of R package. Furthermore, LASSO Cox analysis of R package Gimnet and stepAIC method were used to compress genes. Finally, a formula was built to assess prognosis of CESC samples, as follows:

(1) $$\begin{array}{c} \text{RiskScore}=\overset{n}{\underset{k=0}{\sum }}\beta i\times \text{Expi}, \end{array}$$

where *βi* means the Cox regression coefficient of the *i* gene and Expi means the expression of the *i* gene. Based on median of RiskScore, samples in TCGA-CESC dataset were divided into high-risk group (high group) and low-risk group (low group). The KM survival curve and ROC were used to evaluate the ability to predict prognosis of CESC.

Robustness of the risk model was verified in the TCGA-test dataset, entire TCGA dataset, and GSE44001 dataset.

### 2.10. Nomogram

Whether the RiskScore serve was an independent prediction parameter, univariate and multivariate Cox regression analyses were carried out together with clinicopathological indexes, which were used for developing a nomogram to 1-, 3- and 5-year overall survival (OS) prediction in the “rms” package. For evaluating the nomogram's discriminative ability, ROC analyses concordance index (C-index), and calibration were used.

### 2.11. Statistical Analysis

R software conducted all the statistical analyses (4.1.1). In the study, R packages and tools used were indicated. Statistical analysis methods were detailed in the corresponding sections. *P* < 0.05 was defined as significant (ns, no significance; ^∗∗∗∗^*P* < 0.0001, ^∗∗∗^*P* < 0.001, ^∗∗^*P* < 0.01, and ^∗^*P* < 0.05).

## 3. Results

### 3.1. Genomic Analysis of Oxidative Stress-Related Genes

Firstly, 444 oxidative stress-related genes were acquired from the GSEA website. In TCGA-CESC dataset, 218 of the 291 patients (74.91%) presented oxidative stress-related gene mutations, especially FBXW7 (12%) (Figure 1(a)). The KM survival curve between the mutant sample and nonmutant sample indicated that mutant samples had a better survival time (*P* = 0.037, Figure 1(b)). GSEA analysis revealed that several pathways, such as KRAS_SIGNALING_UP, TNFA_SIGNALING_VIA_NFKB, OXIDATIVE_PHOSPHORYLATION, HYPOXIA, and EPITHELIAL_MESENCHYMAL_TRANSITION, were enriched in the mutant sample (NES > 0, *P* < 0.05, Figure 1(c)).

### 3.2. Identification of Oxidative Stress-Related Gene-Molecular Subtypes

59 oxidative stress-related genes including 35 risk genes (HR > 1) and 24 protect genes (HR < 1) were obtained using univariate Cox survival analysis from 444 oxidative stress-related genes (Figure 2(a)). Pearson's correlation analysis of 59 genes was showed in Figure 2(b). ConsensusClusterPlus analysis indicated that when *k* = 3, 3 clusters, namely, C1, C2, and C3, were determined (Figures 2(c)–2(e)). Oxidative stress scores of the three clusters demonstrated that C2 had the highest scores and C1 had the lowest scores (Figure 2(f)). The KM analysis showed that C3 presented better survival time, followed by C1 and C2 (*P* < 0.0001, Figure 2(g)). Heatmap of 59 gene expressions among the three clusters is showed in Figure 2(h). Clinical feature distribution of the three clusters indicated that survival state (Figure 3(a)) and M stage (Figure 3(f)) had significance (Figures 3(a)–3(g)).

### 3.3. Mutation Characteristics among the Three Clusters

Top 20 mutant genes in the three clusters showed that C3 had higher frequency mutations (42%TTN, 15%FBXW7) vs. C1 (20%TTN, 5%FBXW7) and C2 (25%TTN, 19%FBXW7) (Figure 4(a)). The distributions of fraction altered, number of segments, homologous recombination defects, and tumor mutation burden among the three clusters showed that those characteristics had no significance (Figure 4(b)).

### 3.4. C3 Had Enhanced Tumor Immune Microenvironment

We speculated that subtypes may reflect different immune enrichment. Firstly, the relative abundance of the 28 immune infiltrating cell subpopulations from the TCGA-CESC dataset was visualized by a histogram with ssGSEA, and we observed 27 kinds of immunocytes with significantly different distributions among the three subtypes, and most enriched in C3, such as effector memory CD4+/CD8+ T cells, activated CD4+/CD8+ T cells and natural killer T cells (Figure 5(a)). Our team afterwards evaluated the 10 kinds of immune cell score using MCP-counter methods, and most high enriched in C3 (Figure 5(b)). Everything goes well; C3 sufferers had higher score of StromalScore, ImmuneScore, and ESTIMATEScore (Figures 5(c)–5(e)).

### 3.5. C3 Has Better Response to Immunotherapy

Immune checkpoint inhibitors (ICI) therapy represented by anti-PD-1/L1 agents have undoubtedly greatly promoted antitumor therapy. Therefore, 21 ICI were acquired from HisgAtlas database, and 19 ICI had obviously high expression in C3 than those in C1/C2 (Figure 6(a)). Moreover, the forecasted scores of immune therapy biomarkers were computed via the TIDE arithmetic. Our team assessed the qualities of TIDE, T cell exclusion (exclusion), MDSC, and CAF, which were greater in C2 group versus C1/C3 group, while T cell function disorder scores (dysfunctions) and TAM.M2 were higher in C3 and C1, respectively (Figure 6(b)).

We also explored the susceptible diversity of commonly seen chemo medicines among these 3 groups. The outcomes revealed that the IC_50_ results of cisplatin, erlotinib, sunitinib, paclitaxel, sorafenib, and crizotinib were higher in C1, which unveiled that C1 sufferers were remarkably more susceptible to those medicines (Figure 6(c)).

### 3.6. Coexpression Network of Subtypes Using WGCNA

Using the average linkage method and Pearson's correlation method, a dendrogram of samples (TCGA-CESC) with clinical trait was clustered (Figure 7(a)). The soft-threshold power (*β*) of 5 in TCGA-CESC dataset was estimated to ensure a scale-free network (Figures 7(b) and 7(c)). 13 modules were determined through hierarchical clustering (Figure 7(d)). Furthermore, number genes in 13 modules were calculated; the number of genes in turquoise module is the highest (Figure 7(e)). The correlation analysis between molecular subtypes and 13 modules showed that blue module was positively correlated with C3 (Figure 7(f)). Moreover, module membership and gene significance in the blue module were highly positively correlated (Figure 7(g)). To determine the importance of blue module, ClusterProfiler in R package was used to function enrichment in the blue module. The results showed that tumor-associated pathways, such as cytokine-cytokine receptor interaction, NF-kappa B signaling pathway, Th1 and Th2 cell differentiation, and chemokine signaling pathway, were enriched in the blue module (Figure S1). Thus, the blue module was considered a hub gene module associated to molecular subtype.

### 3.7. Identification of Necroptosis-Related Signature

Six upregulated gene and six downregulated genes associated with CESC prognosis were screened from genes in the blue module using univariate Cox survival analysis in TCGA-CESC training dataset (Figure 8(a)). Based on the characteristics of variable selection and regularization, to fit a generalized linear model, LASSO regression was carried out in hub gene selection for prognostic predicting of high-performance patients (Figures 8(b) and 8(c)). Finally, 5 hub necroptosis genes (GDPD4, TNF, CA9, CX3CL1, and ANGPTL6) were identified (Figure 8(d)). The formula was accordingly constructed as follows: RiskScore = (2.249∗expression level of GDPD4) + (0.336∗expression level of TNF) + (0.204∗expression level of CA9) − (0.217∗expression level of CX3CL1) − (1.832∗expression level of ANGPTL6).

### 3.8. Prognostic Performance Test of Necroptosis-Related Signature

The prognosis-related genes via univariate Cox analysis implicated that CA9, GDPD4, and TNF were risk genes for the prognosis of CESC patients. However, ANGPTL6 and CX3CL1 were protective genes for CESC patients (Figure 9(a)).

Next, RiskScore of patients in TCGA-CESC training dataset was calculated according to the above formula. And then, patients were divided into high RiskScore group and low RiskScore group. The KM survival curve showed that the low group had good performance in OS than in the high group in TCGA-CESC training dataset. The AUCs for 1-year, 3-year, and 5-year survival in the TCGA-CESC training cohort were 0.86, 0.8, and 0.8, respectively (Figure 9(b)). In TCGA-CESC test cohort, samples in low group had better survival time than that in high group, and the AUCs for 1-year, 3-year, and 5-year survival in the TCGA-CESC test cohort were 0.71, 0.69, and 0.73, respectively (Figure 9(c)). In the entire TCGA-CESC cohort, samples in low group had better survival time than that in high group, and the AUCs for 1-year, 3-year, and 5-year survival in the entire TCGA-CESC cohort were 0.78, 0.75, and 0.77, respectively (Figure 9(d)). The similarly results were obtained in the GSE44001 dataset, samples in low group had better survival time than that in high group, and the AUCs for 1-year, 3-year, and 5-year survival in the GSE44001 cohort were 0.62, 0.73, and 0.68, respectively (Figure 9(e)). Of the distributional status of two groups in diverse clinical characteristics (Figures 10(a)–10(g)), remarkable diversity in the three clusters (Figure 10(g)) in TCGA-CESC cohort study were observed. Samples with various clinical characteristics were divided into high group and low group according to RiskScore, and the KM analysis revealed that except N1, M0, and M1, patients in high group had less survival time (Figure 11).

### 3.9. Low Group Had Enhanced Tumor Immune Microenvironment

ssGSEA was used to visualize the relative abundance of 28 immune infiltrating cell subpopulations in high group and low group and observed 10 kinds of immunocytes with significantly different distributions between the high and low group (Figure 12(a)). Ten kinds of immune cells score were evaluated using MCP-counter methods; 6 kinds of immune cells were higher in low group (Figure 12(b)). The low group had higher score of StromalScore, ImmuneScore, and ESTIMATEScore (Figures 12(c)–12(e)).

To observe the relationship between RiskScore and immune function, the correlation analysis between RiskScore and 28 immune cells scores indicated that 28 immune cell scores were negatively associated with RiskScore (Figure 13(a)). R package RSVA for ssGSEA analysis shows the correlation coefficient between functional pathways and RiskScore, and function pathways with correlation coefficient more than 0.2 were selected (Figure 13(b)).

### 3.10. RiskScore and Clinical Pathology Characters Synergistically Predicted the Survival Probability of CESC Patients

The decision tree was constructed according to the age, gender, T stage, stage, grade, and RiskScore in the TCGA-CESC cohort, and the results showed that RiskScore, stage, grade, and T stage were left in the decision tree. As a result, 5 different risk subgroups were identified (Figure 14(a)). The overall survival among the 5 subgroups had significance (Figure 14(b)). Among, patients in risk subgroups C3, C4, and C5 belong to high group, while patients in risk subgroups C1 and C2 belong to low group (Figure 14(c)). In addition, the survival status in the 8 subgroups had significance differences (Figure 14(d)). Univariate and multivariate Cox survival analyses showed that stage, N stage, RiskScore, and T stage were independent prognostic factors (Figures 14(e) and 14(f)). A quantitative method for prognosis prediction of CESC patients was developed through constructing a nomogram based on age, RiskScore, and M stage to predict 1-, 3-, and 5-year CESC overall survival (Figure 14(g)). The calibration curve proved that the prognostic nomogram was reliable and accurate (Figure 14(h)). From decision curve analysis (DCA) and AUC, in clinical decision-making, the RiskScore was found to be able to serve as the most effective prognostic indicator among clinical variables (Figures 14(i) and 14(j)).

### 3.11. Low Group Has Better Response to Immunotherapy

11 ICI had obviously high expression in the low group than those in the high group (Figure 15(a)). The qualities of T cell function disorder scores (dysfunctions), T cell exclusion (exclusion), MDSC, and CAF have differences between the two groups (Figure 15(b)).

Moreover, the IC_50_ results of cisplatin, erlotinib, sunitinib, paclitaxel, sorafenib, and crizotinib were higher in the low group, which unveiled that low group sufferers were remarkably more susceptible to those medicines (Figure 15(c)).

## 4. Discussion

Specifically, based on the oxidative stress-related genes, we determined three molecular subtypes and build a 5-gene signature risk model for the prognosis of CESC, and its validity was further verified in both test, train datasets and GSE44001 dataset. According to the survival analysis, nomogram, and ROC survival risk analysis model, we believe that the model is highly robust. In addition, the risk of CESC was effectively predicted by the model in each clinical subtype of TCGA. We have built a model for prognostic prediction based on oxidative stress genes for the first time.

In our analysis, ANGPTL6 and CX3CL1 were identified as risk factors, and CA9, GDPD4, and TNF were determined as protect factors. Introduced as an angiopoietin-related growth factor, ANGPTL6 has been described as a proangiogenic molecule [27], even though it also serves an essential role in a regulation of energy metabolism [28]. Recently, ANGPTL6 overexpression was associated with tumor proliferation in undifferentiated glioblastoma cells by downregulating miRNA-128 [29]. ANGPTL6 not only facilitates endothelial cell angiogenesis in alpha-fetoprotein- (AFP-) producing gastric cancer but also contributes to the malignancy of the tumor cells themselves [30].

As a seven-transmembrane G-protein-coupled receptor, CX3CR1 mediates the downstream signaling pathway activation via its ligand, CX3CL1 [31]. Various studies have shown that CX3CL1-CX3CR1 interactions are responsible for a variety of clinical diseases, including cancer [32, 33]. Tardáguila et al. [34] revealed the involvement of CX3CL1 in the tumorigenesis of breast cancer. Carbonic anhydrase 9 (CA9), member of the carbonic anhydrase family, is upregulated and regarded as a new potential signer for bladder cancer [35]. TNF-*α*, regulated by circSND1, promotes the migration and invasion of cervical cancer cells [36]. lncRNA LOC105374902/miR-1285-3p/TNF-*α* boosts EMT, migration, and invasion of cervical cancer cells [37]. Up to now, GDPD4 has rarely been reported in tumors. Thus, we speculated that GDPD4 maybe had vital significance for CESC tumorigenesis. Based on the above results, we have reason to believe that these genes are likely to provide clinical prognostic evidence for CESC.

However, this study has some limitations, such as it is necessary for PCR and immunohistochemical verification. Other considerations were not taken into account on our end because the samples lacked essential clinical follow-up information, most notably diagnostic specifics.

## 5. Conclusions

In conclusion, we generated three subgroups based on genes associated with oxidative stress in order to guide tailored therapy for CESC patients and build a 5 oxidative stress-related gene signature for predicting OS. Together, we provided strong preclinical evidence that oxidative stress-related subtypes and RiskScore may be effective for precise treatment of CESC patients.

## Figures and Tables

**Figure 1:** Gene mutation analysis. (a) Single-nucleotide variant of top 20 oxidative stress-related genes. (b) KM survival curve of mutant sample and nonmutant sample. (c) GSEA analysis. ^∗^*P* < 0.05.

**Figure 2:** Identification of molecular subtypes. (a) Univariate Cox survival analysis. (b) Pearson's correlation analysis. (c) Cumulative distribution function. (d) Delta area curve of cumulative distribution function. (e) Heatmap of sample clustering when *k* = 3. (f) The distribution of oxidative stress score in molecular subtypes. (g) KM survival curve of molecular subtypes. (h) Heatmap of oxidative stress-related gene levels in molecular subtypes. ^∗∗∗∗^*P* < 0.0001.

**Figure 3:** The distributions of clinical features: event (a), age (b), grade (c), T stage (d), N stage (e), M stage (f), and stage (g) in molecular subtypes.

**Figure 4:** Genomic analysis. (a) Somatic mutation analysis in molecular subtypes. (b) Analysis of number of segments, tumor mutation burden, fraction altered, and homologous recombination defects in molecular subtypes. ^∗^*P* < 0.05.

**Figure 5:** Tumor immune microenvironment analysis. (a) Analysis of the 28 kinds of immune cells in molecular subtypes. (b) Analysis of the 10 kinds of immune cells in molecular subtypes. (c) Analysis of StromalScore in molecular subtypes. (d) Analysis of ImmuneScore in molecular subtypes. (e) Analysis of ESTIMATEScore in molecular subtypes. ^∗∗∗∗^*P* < 0.0001, ^∗∗∗^*P* < 0.001, ^∗∗^*P* < 0.01, and ^∗^*P* < 0.05.

**Figure 6:** Immunotherapy analysis. (a) The expressions of the 21 immune checkpoints in molecular subtypes. (b) TIDE analysis in molecular subtypes. (c) The box plots of the estimated IC_50_ for cisplatin, erlotinib, sunitinib, paclitaxel, sorafenib, and crizotinib in molecular subtypes. ^∗∗∗∗^*P* < 0.0001, ^∗∗∗^*P* < 0.001, ^∗∗^*P* < 0.01, and ^∗^*P* < 0.05.

**Figure 7:** WGCNA. (a) Sample clustering tree. (b) Various soft-thresholding powers were applied in the analysis of the scale-free fit index (*β*). (c) Various soft-thresholding powers were applied in the analysis of the mean connectivity. (d) Based on a dissimilarity measure, a dendrogram on all differentially expressed genes clustered (1-TOM) was shown. (e) Number of genes in 13 modules. (f) The correlation analysis between the three subtypes and 13 modules. (g) Correlation analysis between gene significance in C3 and blue module membership.

**Figure 8:** Identification of promising candidates. (a) Potential promising candidates were screened through the survival analysis of the genes of blue module. (b) The coefficients of various promising candidates. (c) A confidence interval under lambda. (d) Five promising genes were identified.

**Figure 9:** Prognostic ability of oxidative stress-related gene signature. (a) A forest map showed 5 oxidative stress-related gene signature identified by Cox proportional hazard regression. (b) KM survival and ROC of 5 necroptosis-related gene signature in the training cohort. (c) KM survival and ROC of 5 necroptosis-related gene signature in the test cohort. (d) KM survival and ROC of 5-gene signatures in the entire TCGA cohort. (e) KM survival and ROC of 5-gene signatures in the GSE44001 cohort.

**Figure 10:** The distribution of RiskScore in patients with (a) age, (b) T stage, (c) N stage, (d) M stage, (e) Stage, (f) gender, and (g) clusters.

**Figure 11:** KM prognosis curve of high group and low group in samples with (a) age > 45, (b) age < 45, (c) T1+T2 stage, (d) T3+T4 stage, (e) N0 stage, (f) N1 stage, (g) M0 stage, (h) M1 stage, (i) stage I+II, (j) stage III+IV, (k) G1+G2, and (l) G3.

**Figure 12:** Tumor immune microenvironment analysis. (a) Analysis of the 28 kinds of immune cells between high group and low group. (b) Analysis of the 10 types of immune cells between the low and high groups. (c) Analysis of StromalScore between the low and high groups. (d) Analysis of ImmuneScore between the low and high groups. (e) Analysis of ESTIMATEScore between the low and high groups. ^∗∗∗∗^*P* < 0.0001, ^∗∗∗^*P* < 0.001, ^∗∗^*P* < 0.01, and ^∗^*P* < 0.05.

**Figure 13:** Functional enrichment analysis. (a) The correlation analysis between the 28 kinds of immune cells and RiskScore. (b) The correlation analysis between the KEGG pathways and RiskScore.

**Figure 14:** RiskScore and clinical pathology characters could synergistically predict CESC survival rate. (a) 5 different risk subgroups were identified. (b) The overall survival among 5 subgroups had significance. (c) Patients in risk subgroups C3, C4, and C5 belong to high group, while patients in risk subgroups C1 and C2 belong to low group. (d) The survival status in 5 subgroups had significance differences. (e, f) Univariate and multivariate Cox survival analyses. (g) AUC analysis. (h) A prognostic nomogram based on stage, N stage, T stage, and RiskScore to predict 1-, 3-, and 5-year OS of CESC patients. (i) Calibration curve supported the reliability and the accuracy of the prognostic nomogram. (j) Decision curve analysis (DCA) validated the RiskScore as the most effective indicator compared with other clinical variables in the clinic. ^∗^*P* < 0.05, ^∗∗^*P* < 0.01, and ^∗∗∗^*P* < 0.001.

**Figure 15:** Immunotherapy analysis and drug analysis of the high group and low group. (a) The expressions of 21 immune checkpoints between the high group and low group. (b) TIDE analysis between the low and high groups. (c) Box plots on the estimated IC_50_ for erlotinib, sunitinib, cisplatin, sorafenib, paclitaxel, and crizotinib between the low and high groups. ^∗^*P* < 0.05, ^∗∗^*P* < 0.01, ^∗∗∗^*P* < 0.001, and ^∗∗∗∗^*P* < 0.0001.

**Table 1:** Clinical information of sample in datasets.

Clinical features	TCGA-CESC	GSE44001
OS		
0	220	262
1	71	38
T stage		
T1	137	
T2	67	
T3	16	
T4	10	
TX	61	
N stage		
N0	128	
N1	55	
NX	108	
M stage		
M0	107	
M1	10	
MX	174	
Stage		
I	159	
II	64	
III	41	
IV	21	
X	6	
Grade		
G1	18	
G2	129	
G3	116	
G4	1	
GX	27	
Age		
≤45	139	
>45	152	

## Data Availability

The dataset analyzed in this study could be found in GSE44001 at https://www.ncbi.nlm.nih.gov/geo/query/acc.cgi?acc=GSE44001.

## Supplementary Materials

Supplementary Materials Figure S1: function enrichment analysis. (A) BP of GO analysis. (B) CC of GO analysis. (C) MF of GO analysis. (D) KEGG analysis.
